The article "Knockout of circRNA single stranded interacting protein 1 (circRBMS1) played a protective role in myocardial ischemia-reperfusion injury though inhibition of miR-2355-3p/Mammalian Sterile20-like kinase 1 (MST1) axis" was retracted in 2026. Reasons: concerns about the data; concerns about the results or conclusions.

# Knockout of circRNA single stranded interacting protein 1 (circRBMS1) played a protective role in myocardial ischemia-reperfusion injury though inhibition of miR-2355-3p/Mammalian Sterile20-like kinase 1 (MST1) axis

**DOI:** 10.1080/21655979.2022.2068896

**Published:** 2022-05-25

**Authors:** Yingping Liang, Huanhuan Jie, Qin Liu, Chang Li, Renjie Xiao, Xianliang Xing, Jing Sun, Shuchun Yu, Yanhui Hu, Guo-hai Xu

**Affiliations:** Department of Anesthesiology, Second Affiliated Hospital of Nanchang University, Nanchang, China

**Keywords:** Myocardial I/R injury, circRBMS1, miR-2355-3p, MST1

## Abstract

Evidence suggests circRBMS1 regulates mRNA to mediate cell apoptosis, inflammation, and oxidative stress in different diseases. MST1 is reported to be the target and activator of apoptosis-related molecules and signaling pathways. Hence, the present study aims to investigate the role of circ-RBMS1/miR-2355-3p/MST1 in the development of I/R injury. *In vitro* experiments showed increased circ-RBMS1 and decreased miR-2355-3p in H/R-induced HCMs. CircRBMS1 served as a sponge for miR-2355-3p and miR-2355-3p targeted MST1. Furthermore, knockout of circRBMS1 attenuated cell apoptosis, oxidized stress, and inflammation in H/R-induced HCMs. *In vivo* experiments indicated circRBMS1 knockdown attenuated cardiac function damage, cell apoptosis, oxidative stress injury and inflammatory response through miR-2355-3p/MST1 axis in mice. In summary, these results demonstrated circRBMS1 played a protective role in myocardial I/R injury though inhibition of miR-2355-3p/MST1 axis. It might provide a new therapeutic target for cardiac I/R injury.

## Highlights

- circRBMS1 was increased and miR-2355-3p was decreased in H/R induced HCMs.
- circRBMS1 knockdown attenuated H/R induced suppression of cell viability, and aggravation of cell apoptosis, oxidative stress and inflammation in HCMs.
- circRBMS1 mediated H/R induced cell injury by targeting miR-2355-3p/MST1 axis.
- circRBMS1 knockdown attenuated impaired cardiac performance, cell apoptosis, oxidative stress injury and inflammation response through regulating miR-2355-3p/MST1 axis in I/R mouse model.

## Introduction

Cardiovascular diseases, such as ischemic heart disease and stroke, account for a quarter of the internationally death of more than 13 million people every year [1]. Though myocardial reperfusion is of great importance for treating ischemic myocardium caused by coronary occlusion, initial ischemia followed with reperfusion may lead to cardiac tissue damage, namely cardiac I/R injury [2]. Emerging evidence shows cardiac I/R injury suggests an aggravation for myocardial cell injury and it has identified as a vital risk factor for cardiovascular diseases [3]. Hence, it’s very essential to study the mechanism of I/R-induced cardiac cell injury to prevent cardiovascular diseases.

The article "Knockout of circRNA single stranded interacting protein 1 (circRBMS1) played a protective role in myocardial ischemia-reperfusion injury though inhibition of miR-2355-3p/Mammalian Sterile20-like kinase 1 (MST1) axis" was retracted in 2026. Reasons: concerns about the data; concerns about the results or conclusions.

Cell proliferation and apoptosis are essentially biological process involved in the pathological mechanism of ischemic myocardium [4]. Oxidative stress mediates cell apoptosis, inflammatory response, and lipid peroxidation to regulate pathological process of I/R injury [5]. As reported, inflammation triggers unbalanced expression of inflammatory mediators, which in turn aggravates inflammation and ischemic injury [6]. Increasing evidence indicates various circRNAs are associated with the pathogenesis of multiple cardiovascular diseases, for instance, ischemia reperfusion injury, myocardial infarction, coronary artery disease, heart failure, and so on [7]. heart-related circRNA (CircHRCR) functions as a sponge of miR-223 to alleviate cardiac injury, suggesting an attractive therapeutic target for the treatmennt of heart failure [8]. Circular RNA ciRS‐7 (ciRS-7) is reported to suppress cell proliferation, invasion, and tube formation as well as promote cell apoptosis through sponging miR-26a-5p via PI3K/AKT and JNK/p38 signaling pathways in human microvascular endothelia, indicating the function of ciRS-7 in miocardial infarction [9]. Interesting, a previous study reports circRBMS1 mediates cell apoptosis, inflammation, and oxidative stress in chronic obstructive pulmonary disease [10]. Close association is found between miR-2355-3p and various diseases, such as diabetic nephropathy [11], pancreatic cancer [12] and heart failure [13]. MST1 serves as the target and activator of apoptosis-related molecules and signaling pathways, regulating neuronal cell apoptosis or microglia activation in myocardial and brain injury [14]. Nevertheless, no researches illustrate the functions and regulating relationship of circRBMS1, miR-2355-3p, and MST1 in cell apoptosis, inflammatory response, and oxidative stress in myocardial I/R injury.

Bioinformatics analysis indicates circRBMS1 binds to miR-2355-3p and MST1 is the predicted target of miR-2355-3p. Thus, we hypothesized the regulating among circRBMS1, miR-2355-3p, and MST1 might affect the pathogenesis and development of myocardial I/R injury. This study aims to investigate the role and the regulation among circRBMS1, miR-2355-3p, and MST1 in myocardial I/R injury. Our *in vivo* and *in vitro* studies illustrate circRBMS1 mediates cell viability, apoptosis, oxidative stress, and inflammatory response in myocardial I/R injury by targeting miR-2355-3p/MST1 axis.

## Methods

### Cell culture and H/R-induced cell injury

Primary human cardiac myocytes (HCMs, ATCC) were cultured in RPMI-1640 containing 10% FBS, 100 μg/mL streptomycin, and 100 U/mL penicillin (MedChemExpress LLC) at 37°C with 95% air and 5% CO_2._

To establish the model of H/R-induced cell injury, HCMs were cultured in a hypoxia chamber with an anerobic pouch under 5%CO_2_/95%N_2_ for 24 h followed with reoxygenation at 37°C with 5% CO_2_ for 3 h.

The article "Knockout of circRNA single stranded interacting protein 1 (circRBMS1) played a protective role in myocardial ischemia-reperfusion injury though inhibition of miR-2355-3p/Mammalian Sterile20-like kinase 1 (MST1) axis" was retracted in 2026. Reasons: concerns about the data; concerns about the results or conclusions.

### Cell transfection

miR-2355-3p vector (mimics or inhibitor) and NC controls (50 nM) were purchased from GenePharm (Athens, Greece). CircRBMS1 knockdown vector (sh-circRBMS1, 100 nM) and NC vector (sh-NC) was purchased and synthesized by GenePharm. Cells were cultured in serum-free Opti-MEM medium, followed with 48 h transfection of miRNAs and plasmids using Lipofectamine 2000 (Invitrogen).

### CCK-8 assay

The detection of cell viability of HCMs and myocardial tissues were conducted using CCK-8 assay. In brief, cells were placed in 96‐well plates (3 × 10^3^/well) overnight. At 48 h after transfection, each well was supplemented with 10 μL of CCK-8 solution. At 2 h after the incubation, the absorbance of samples were determined at 490 nm using a microplate reader (Molecular Devices).

### TUNEL assay

Myocardial tissues or HCMs were collected and stained with DAPI. Cell apoptosis was analyzed using a Roche Apoptosis Detection Kit. Apoptotic rate was identified as TUNEL positive cells to total cells. Images were taken using fluorescence microscopy (Leica Microsystems).

### Evaluation of oxidative stress

Contents of superoxide dismutase (SOD) and malondialdehyde (MDA) in HCMs and mouse serum were detected using commercial kits: SOD assay kit (A001-3-1) and microscale MDA assay kit (A003-2-2, Nanjing Jiancheng Bioengineering institute).

Reactive oxygen species (ROS) generation was detected using Immunofluorescence assay. Cells were fixed with 4% formaldehyde followed with washing using iced PBS for three times. Subsequently, PBS with 0.25% Triton X-100 was used for cell permeabilization followed with washing by iced PBS for three times. Cells were incubated with primary polyclonal rabbit anti‑human ROS antibody (LS-C328570, 1/10, LSBio) at 4°C overnight. The samples were supplemented with polyclonal goat anti‑human IgA secondary antibody (LS‑C60498, 1/1000, LSBio) and incubated for 2 h at room temperature. Afterward, the collected samples were mounted and imaged by a confocal microscope.

### ELISA

Expressions of TNF-α, IL-1β, and IL-6 in cell supernatants and myocardial tissue were detected using ELISA assay. Commercial kits were used for the detection, including Human TNF-α ELISA Kit (ab46087, range: 25 pg/mL~800 pg/mL), Mouse TNF-α ELISA Kit (ab100747, range: 93.75 pg/mL~6000 pg/mL), Human IL-1β ELISA Kit (ab214025, range: 14.06 pg/mL~900 pg/mL), Mouse IL-1β ELISA Kit (ab197742, 1.56 pg/mL~100 pg/mL), Human IL-6 ELISA Kit (ab229434, range: 0.97 pg/mL~2000 pg/mL), and Mouse IL-6 ELISA Kit (ab46100, range: 15.6 pg/mL~500 pg/mL). All the kits were purchased from Abcam.

The article "Knockout of circRNA single stranded interacting protein 1 (circRBMS1) played a protective role in myocardial ischemia-reperfusion injury though inhibition of miR-2355-3p/Mammalian Sterile20-like kinase 1 (MST1) axis" was retracted in 2026. Reasons: concerns about the data; concerns about the results or conclusions.

### Western blot

Total proteins were collected from lysed HCMs. Equal amounts of the samples were isolated by 12% SDS-PAGE and transferred onto PVDF membranes, blocking with 5% defatted milk. The protein samples were then incubated with primary antibodies at 4°C overnight followed with incubation of secondary antibody goat anti-rabbit IgG H&L preadsorbed (ab96899, 1/1000) at 37°C for 45 min. Primary antibodies including Cleaved Caspase-3 antibody (ab2302, 1/50), Bax antibody (ab182733, 1/2000), Bcl-2 antibody (ab182858, 1/2000) and MST1 antibody (ab245190, 1/1000). All the antibodies were obtained from Abcam. β-actin was used as a control. Protein bands were visualized by Chemiluminescence reagents (Cell Signaling Technology) and quantified by Image-Pro plus software 6.0.

### Luciferase reporter assay

circRBMS1 3’‐UTR or MST1 3’‐UTR with/without the predicted responsive element of miR-2355-3p (circRBMS1-WT, circRBMS1-MUT, MST1-WT, and MST1-MUT) were amplified and inserted into pGL3 vector (Hunan Fenghui Biotechnology Co., Ltd). Samples were transfected with luciferase reporter vectors and miR-2355-3p mimics or NC control (Biomics Biotech) using Lipofectamine 2000 (Invitrogen). At 48 h after the transfection, the luciferase activity was analyzed using a TransDetect® Double-Luciferase Reporter Assay Kit (FR201-01, TransGen Biotech Co., Ltd.) and normalized to value of Renilla luciferase activity.

### RNA pull‐down assay

The biotinylated circRBMS1 probe with oligo probe (RiboBio) as the control was incubated with streptavidin magnetic beads (Cat. No. HY-K0208, MedChemExpress) at room temperature for 2 h. HCMs (1 × 10^7^) were lysed and mixed with circRBMS1 probe or oligo probe at 4°C overnight. Subsequently, the extraction of bound RNA was conducted using Trizol and detection of RNA was performed using RT-PCR.

### qRT‐PCR

Levels of miR-2355-3p, circRBMS1, and MST1 were detected using qRT‐PCR. Extraction of total RNA from HCMs and tissues were conducted by TRIzol reagent (Invitrogen). For miR-2355-3p quantification, 2 μg of template RNA was reversely transcribed into cDNA using TransScript First-Strand cDNA Sythesis SuperMix. The fluorescence quantitative PCR reaction was performed on Thermal Cycler Dice Real-Time System II (Takara). For quantification of circRBMS1 or MST1, Prime-Script™ One Step RT-qPCR kit (Takara) was applied for reverse transcription from RNA into cDNA. The PCR reactions were performed on an ROX Reference Dye II (GenStar) on StepOnePlusTM Real-Time PCR System (Applied Biosystems). The primer sequences used in qPCR were as follows: U6 forward 5'-CTCGCTTCGGCAGCACA-3' and reverse 5'- AACGCTTCACGAATTTGCGT-3'; GAPDH forward 5'-CACCAGGGCTGCTTTTAACTC-3’ and reverse 5'-TGGAAGATGGTGATGGGATTT-3'; miR‐2355‐3p forward 5'-CTGAGGGATCCCCAGATACAATGG-3' and reverse 5'-GTGCAG GGTCCGAGGT-3'; circ-RBMS1: forward 5'-CCCTGATCTCCATACCCAGA-3' and reverse 5'-TGGAGTCGAGTGTTTGCAGT-3'; MST1 forward 5'-AGACCTCCAGGAGATAATCAAAGA-3' and reverse 5'-AGATACAGAACCAGCCCCACA-3'. The expression of mRNA and miRNA was normalized to GAPDH and U6, respectively. Quantification of RNA was analyzed using 2^−ΔΔCt^ method.

The article "Knockout of circRNA single stranded interacting protein 1 (circRBMS1) played a protective role in myocardial ischemia-reperfusion injury though inhibition of miR-2355-3p/Mammalian Sterile20-like kinase 1 (MST1) axis" was retracted in 2026. Reasons: concerns about the data; concerns about the results or conclusions.

### Myocardial I/R injury mouse model

A total of 40 eight-week male C57BL/6 mice (20 ~ 26 g) were randomly divided into the following 5 groups: 1) Control; 2) Sham group; 3) I/R group; 4) I/R+ sh-NC group; 5) I/R+ sh-circRBMS1 group (n = 8 for each group). Surgery was performed as previously reported [15]. 2% isoflurane inhalation was used for mice anesthesia, accompanied by artificial ventilation (80 strokes/minute). The exposure of heart as well as left anterior descending artery (LAD) at the fourth intercostal space was performed by thoracotomy. Subsequently, LAD was ligated using a 7–0 silk suture. The reperfusion was performed 45 min later and last for 3 h.

The construction of adenoviruses vectors to inhibit circRBMS1 was conducted (lenti-sh-circRBMS1) and lenti-sh-circRBMS1 or lenti-sh-NC (100 μl) was injected through tail vein. The following experiments were performed 5 days after adenovirus administration. This study obeyed international guidelines for animal research projects and obtained the approval from the Animal Ethics Committee of Second Affiliated Hospital of Nanchang University.

### Enzyme activity detection

Briefly, a total of 10 μL serum samples were collected from I/R mice or the sham. Serum indexes of myocardial infarction were determined using commercial kits: LDH assay kit (A020-2-2, OD: 450 nm), CK assay kit (A032-1-1, OD: 660 nm) and CK-MB assay kit (H197-1-2, OD: 660 nm. All from Nanjing Jiancheng Bioengineering institute).

### Echocardiographic assessment

Ejection fraction (LVEF), LV internal diameter systolic (LVIDS), and LV end-diastolic diameter (LVIDd) were recorded to assess the cardiac function indicators. Calculation of fractional shortening of LV fractional shortening (LVFS) was conducted using the formula: LVFS = [(LVIDd/LVIDs)/LVIDd] × 100%.

### Data analysis

All data were displayed as mean ± standard deviation (SD). Comparison for two groups was made by the Student’s *t* test. The analysis and graph of all data were conducted using Graphpad Prism 6.0 software. It was considered to be significance when *P* < 0.05. All experiments were performed at least three times.

The article "Knockout of circRNA single stranded interacting protein 1 (circRBMS1) played a protective role in myocardial ischemia-reperfusion injury though inhibition of miR-2355-3p/Mammalian Sterile20-like kinase 1 (MST1) axis" was retracted in 2026. Reasons: concerns about the data; concerns about the results or conclusions.

## Results

Bioinformatics analysis indicated the target relationship between circRBMS1 and miR-2355-3p, as well as MST1 and miR-2355-3p. Previous studies showed circRBMS1, miR-2355-3p, and MST1 was associated with I/R injury. Thus, we hypothesized the regulating relationship among circRBMS1, miR-2355-3p, and MST1 might affect the pathogenesis and development of myocardial I/R injury. This study conducted *in vivo* and *in vitro* experiments to investigate the functions and the regulation among circRBMS1, miR-2355-3p, and MST1 for cell apoptosis, cell viability, oxidative stress, and inflammation in myocardial I/R injury. Our findings indicated knockout of circRBMS1 played a protective role in myocardial I/R injury though inhibition of miR-2355-3p/MST1 axis.

### Knockdown of circRBMS1 attenuated H/R-induced cell injury

A H/R-induced cell model was established to investigate the role of circRBMS1 in myocardial I/R injury. CircRBMS1 expression was elevated about 3 times in H/R-induced HCMs and was decreased around 4 times by sh-circRBMS1 transfection (Figure 1a-b). CCK-8 assay showed circRBMS1 knockdown rescued H/R-induced inhibition for cell viability (Figure 1c). CircRBMS1 knockdown also reduced H/R-induced elevation of TUNEL positive cells (Figure 1d). Besides, downregulated circRBMS1 suppressed protein expressions of cleaved-caspase 3 and Bax, but increased Bcl-2 expression, suggesting inhibition of circRBMS1 alleviated cell apoptosis in H/R-induced HCMs (Figure 1e). ROS production was decreased by circRBMS1 interference (figure 1f). Additionally, decreased MDA content and increased SOD expression were also observed in H/R-induced HCMs transfected with sh-circRBMS1 (Figure 1g-h). Data showed descended levels of TNF-α, IL-1β, and IL-6 in H/R-induced cells transfected with sh-circRBMS1. All the findings suggested that circRBMS1 knockdown enhanced cell viability, and suppressed cell apoptosis, oxidative stress, and inflammatory response in H/R-induced HCMs.

**Figure 1.** Knockdown of circRBMS1 attenuated H/R-induced cell injury. (a-b) qRT-PCR analysis of circRBMS1 expression. H/R-induced HCMs were transfected with sh-RBMS1 or sh-NC. (c) CCK-8 assay for cell viability. (d) TUNEL assay for cell apoptosis. Scale bars: 50 μm. (e) Western blot analysis of cleaved-caspase 3, Bax and Bcl-2. (f) ROS generation was detected using immunofluorescence assay. Scale bars: 100 μm. (g-h) Detection of MDA contents and SOD level. (i-k) ELISA data of TNF-α, IL-1βand IL-6. **P < 0.01 compared with control or H/R+ sh-NC.

The article "Knockout of circRNA single stranded interacting protein 1 (circRBMS1) played a protective role in myocardial ischemia-reperfusion injury though inhibition of miR-2355-3p/Mammalian Sterile20-like kinase 1 (MST1) axis" was retracted in 2026. Reasons: concerns about the data; concerns about the results or conclusions.

### circRBMS1 served as a sponge for miR-2355-3p

The regulation between miR-2355-3p and circRBMS1 was investigated. Bioinformatics analysis showed circRBMS1 was predicted to target miR-2355-3p (Figure 2a). Compared with the control group, miR-2355-3p expression was increased 19 times in miR-2355-3p minics group (Figure 2b). Additionally, the luciferase intensity of circRBMS1-WT was reduced by miR-2355-3p overexpression (Figure 2c), suggesting that miR-2355-3p acted as a functionally direct target for circRBMS1. The targeting relationship was further confirmed in the analysis of pull-down assay (Figure 2d). Additionally, H/R-induced donwregulation of miR-2355-3p could be enhanced by sh-circRBMS1 (Figure 2e). Taking together, circRBMS1 acted as a sponge of miR-2355-3p in H/R-induced HCMs.

**Figure 2.** CircRBMS1 targeted miR-2355-3p. (a) circRBMS1 was predicted to bind to miR-2355-3p (Starbase). (b) qRT-PCR determined miR-2355-3p expression in HCMs transfected with miR-2355-3p mimics, NC mimics or the control. (c) Detection of luciferase activity. (d) Pull-down assay showed elevated enrichment of miR-2355-3p in HCMs transfected with biotin-labeled circRBMS1. (e) qRT-PCR analysis for miR-2355-3p expression. **P < 0.01 compared with control, miR-NC, bio-NC or H/R+ sh-NC.

### Elevated miR-2355-3p alleviated H/R-induced cell injury

The function of miR-2355-3p was studied in H/R-induced cell injury. Suppressed cell viability in H/R-induced cells was obviously activated by miR-2355-3p mimics (Figure 3a). Apoptotic ratio of cells was increased by H/R treatment and decreased approximately 3 folds by miR-2355-3p overexpression (Figure 3b). Enhanced ROS production induced by H/R treatment was reduced around four folds by miR-2355-3p mimics (Figure 3c). Besides, H/R-induced activation of pro-inflammatory mediators were inhibited by miR-2355-3p mimics (FIG D). These data illustrated miR-2355-3p overexpression attenuated cell apoptosis, ROS generation, and inflammation in cardiac myocytes.

**Figure 3.** Elevated miR-2355-3p alleviated H/R-induced cell injury. (a) CCK-8 assay results of cell viability in Control, H/R, H/R+ miR-NC, and H/R+ miR-2355-3p. (b) TUNEL assay analyzed cell death. Scale bars: 50 μm. (c) ROS generation was analyzed using immunofluorescence assay. Scale bars: 100 μm. (d) ELISA detection for TNF-α, IL-1β and IL-6. **P < 0.01 compared with miR-NC, bio-circRBMS1 or H/R+ sh-circRBMS1.

### circRBMS1 mediated H/R-induced cell injury by targeting miR-2355-3p/MST1 axis

The underlying molecular mechanism of circRBMS1 was further studied. Bioinformatics analysis predicted the potential-binding site between miR-2355-3p and MST1 (Figure 4a). The luciferase intensity of MST1-WT was decreased about four folds by miR-2355-3p mimics, whereas no obvious change was found for that of MST1-MUT (Figure 4b). In addition, miR-2355-3p mimics exhibited inhibition on MST1 expression (Figure 4c). The expression of miR-2355-3p was successfully knockdown by miR-2355-3p inhibitor (Figure 4d). It also found upregulated MST1 in H/R-induced cells could be downregulated by sh-circRBMS1, which was reversed by the inhibition of miR-2355-3p (Figure 4e). Compared with NC group, an around 2-fold increase of cell viability was observed in sh-circRBMS1 group, while, miR-2355-3p inhibitor notably suppressed cell viability enhanced by sh-circRBMS1 (figure 4f). Interestingly, the contrary result was observed on cell apoptosis (Figure 4g). MRNA and protein levels of apoptotic genes were analyzed to further confirm the function of circRBMS1 and miR-2355-3p for cell apoptosis. The results illustrated sh-circRBMS1 exhibited inhibition on pro-apoptotic genes and promotion on anti-apoptotic gene, nevertheless, the effects could be reversed by miR-2355-3p inhibitor (Figure 4h). Moreover, ROS generation (Figure 4i) and inflammatory response (Figure 4j-l) were markedly suppressed by sh-circRBMS1, the results of which were rescued by miR-2355-3p knockdown. The above findings suggested that circRBMS1 mediated H/R-induced cell injury through targeting miR-2355-3p/MST1 axis.

The article "Knockout of circRNA single stranded interacting protein 1 (circRBMS1) played a protective role in myocardial ischemia-reperfusion injury though inhibition of miR-2355-3p/Mammalian Sterile20-like kinase 1 (MST1) axis" was retracted in 2026. Reasons: concerns about the data; concerns about the results or conclusions.

**Figure 4.** CircRBMS1 mediated H/R-induced cell injury by targeting miR-2355-3p/MST1 axis. I/R induced HCMs were transfected with sh-NC, sh-circRBMS1 or sh-circRBMS1 and miR-2355-3p inhibitor. (a) Predicted binding site for miR-2355-3p and MST1. (b) Detection of luciferase activity. (c) MST1 protein was determined. (d) Detection of miR-2355-3p was conducted using qRT-PCR. (e) Western blot for MST1 quantification. (f) Assessment of cell viability. (g) Calculation of TUNEL positive cells. Scale bars: 50 μm. (h) Western blot for cleaved-caspase 3, Bax and Bcl-2. (i) ROS generation was detected using immunofluorescence assay. Scale bars: 100 μm. (j-l) ELISA results for the contents of TNF-α, IL-1β and IL-6. *P < 0.05, **P < 0.01 compared with control, miR-NC, H/R+ sh-NC or H/R+ sh-circRBMS1+ anti-miR-2355-3p.

### circRBMS1 knockdown mediated myocardial I/R injury by regulating miR-2355-3p/MST1 axis in mice

Finally, a I/R mouse model was established to confirm the regulating mechanism of circRBMS1 *in vivo*. No obvious difference was found for the structure and inflammation in myocardial tissue between the control and sham group (Figure 5a). Hence, the sham group was studied in the following experiments. The activity of serum enzyme including LDH, CK, and CK-MB was activated in I/R-induced mice but inhibited by sh-circRBMS1 (Figure 5b). Echocardiographic parameters analysis revealed decreased levels of LVEF and LVFS in I/R mice was elevated by sh-circRBMS1 (Figure 5c), indicating sh-circRBMS1 played a protective role for heart function in I/R mice. Swollen and necrotic cardiomyocytes with disordered arrangement of myocardial bundles were observed in myocardial tissue collected from I/R mice, however, sh-circRBMS1 significantly attenuated structural damage in myocardial tissue (Figure 5d). PCR quantification of circRBMS1 and MST1 was increased in I/R mice but reduced by inhibition of circRBMS1. In contrast, miR-2355-3p expression was reduced in I/R mice but increased by sh-circRBMS1 (Figure 5e-f). Compared to the sham group, the ratio of TUNEL positive cell was elevated in myocardial tissue of I/R group, but reduced by sh-circRBMS1, suggesting sh-circRBMS1 alleviated cell apoptosis in I/R mice (Figure 5g). Besides, increased serum contents of MDA and reduced SOD were found in I/R mice, however, the contents of which were decreased by sh-circRBMS1, namely, sh-circRBMS1 attenuated oxidative stress in I/R mice (Figure 5h). The activated inflammatory mediator (TNF-α, IL-1Β, and IL-6) were suppressed by sh-circRBMS1 (Figure 5i). These results illustrated that circRBMS1 knockdown attenuated the damage of cardiac function, cell apoptosis, oxidative stress injury, and inflammatory response by mediating miR-2355-3p/MST1 axis in I/R mice.

The article "Knockout of circRNA single stranded interacting protein 1 (circRBMS1) played a protective role in myocardial ischemia-reperfusion injury though inhibition of miR-2355-3p/Mammalian Sterile20-like kinase 1 (MST1) axis" was retracted in 2026. Reasons: concerns about the data; concerns about the results or conclusions.

**Figure 5.** circRBMS1 knockdown mediated myocardial I/R injury by regulating miR-2355-3p/MST1 in mice. The I/R mouse model was established. (a) H&E staining for myocardial tissue in control and sham group. Scale bars: 100 μm. (b) The mice were grouped: Sham, I/R, I/R+ lenti-sh-NC and I/R+ lenti-sh-circRBMS1. Enzyme activity of LDH, CK and CK-MB. (c) Echocardiographic parameters LVEF and LVFS were recorded. (d) H&E staining for myocardial tissue. Scale bars: 100 μm. Swollen and necrotic cardiomyocytes and disordered arrangement of myocardial bundles were observed in myocardial tissue of I/R-induced mice, conversely, sh-circRBMS1 significantly attenuated structural damage of myocardial tissue. (e) qRT-PCR analysis of circRBMS1. (f) qRT-PCR analysis of miR-2355-3p and MST1. (g) TUNEL assay for cell apoptosis. Compared to the sham group, ratio of TUNEL positive cell was increased in myocardial tissue of I/R group, while sh-circRBMS1 reduced the ratio of TUNEL positive cell in I/R group. (h) Detection of serum levels of MDA and SOD. (i) ELISA data for serum TNF-α, IL-1β and IL-6. *P < 0.05, **P < 0.01 compared with sham or H/R+ sh-NC.

## Discussion

Accumulating evidences reveal cell apoptosis, inflammatory response, and oxidative stress play important roles in myocardial I/R injury [16,17]. Nevertheless, the underlying molecular mechanism of I/R injury still remains unclear. This study conducted *in viv*o and *in vitro* experiments to investigate the role of miR-2355-3p, circRBMS1, and MST1 in mediating cell viability and apoptosis, oxidative stress and inflammatory response in myocardial I/R injury.

The article "Knockout of circRNA single stranded interacting protein 1 (circRBMS1) played a protective role in myocardial ischemia-reperfusion injury though inhibition of miR-2355-3p/Mammalian Sterile20-like kinase 1 (MST1) axis" was retracted in 2026. Reasons: concerns about the data; concerns about the results or conclusions.

CircRNAs possess different binding site of miRNAs and act as the sponge for specific miRNA [18]. As reported, the expression of circRNA tetratricopeptide repeat domain 3 (circ-Ttc3) was notably elevated in hypoxia-induced cardiomyocytes. Functional research demonstrated circ-Ttc3 regulated adenosine triphosphate (ATP) expression and cell apoptosis by sponging miR-15b-5p in cardiomyocytes, suggesting a protective effect of circ-Ttc3 on myocardial infarction [19]. CircRNA Zinc finger 644 (Circ-Zfp644) enhanced the expression of pro-fibrotic mediator LIM kinase-1 (LIMK1) through sponging miR-93-5p in *in vitro* model of cardiac hypertrophy [20]. miR-383 enhanced steroidogenesis by targeting RBMS1 via c-Myc activation in mouse ovarian granulosa cells [21]. RBMS1 was reported to be a target of miR-106b. Reduced expression of RBMS1 was observed in prostate tumors and PCa cell lines, and RBMS1 showed inhibiting effect on PCa cell proliferation, suggesting RBMS1 acted as a tumor suppressor [22]. A previous study found circRBMS1 expression was increased in patients with chronic obstructive pulmonary disease. The *in vitro* study further illustrated that inhibition of circ-RBMS1 attenuated cell apoptosis, inflammatory response and oxidative stress in 16HBE cells exposed to cigarette smoke [10]. Our findings also suggested circRBMS1 served as a sponge for miR-2355-3p in HCMs. Moreover, knockout of circ-RBMS1 attenuated myocardial I/R injury by regulating miR-2355-3p/MST1 axis in H/R-induced cell model and I/R mice model.

Numerous studies indicate miR-2355-3p is associated with biological progression of various diseases. miR-2355-3p expression was decreased in diabetic rats. Research on molecular mechanism illustrated long noncoding RNA metastasis-associated lung adenocarcinoma transcript 1 (lncRNA MALAT1) mediated diabetic nephropathy by sponging miR-2355-3p/IL6ST axis [11]. Another study also reported elevated miR-2355-3p enhanced AK4 expression, and miR-2355-3p/DDX3X/AK4 axis was involved in proliferation and invasion of pancreatic cancer cells [12]. Clinic data showed an obvious upregulation of miR-2355-3p in patients with lung adenocarcinoma. Furthermore, cell model revealed that miR-2355-3p inhibited progression of lung adenocarcinoma by targeting zinc finger CCHC-type containing 14 (ZCCHC14), indicating miR-2355-3p might become a potential biomarker for the diagnosis of lung adenocarcinoma [23]. Liang et al. reported that lncRNA Sox2 overlapping transcript (SOX2-OT) knockdown attenuated cell apotheosis, inflammation, and oxidative stress through regulating miR-2355-3p expression in rats with heart failure [13]. In this study, we for the first time described reduced miR-2355-3p in H/R-induced HCMs, besides, overexpression of miR-2355-3p was able to alleviate H/R-induced cell apoptosis, oxidative stress, and inflammation.

The article "Knockout of circRNA single stranded interacting protein 1 (circRBMS1) played a protective role in myocardial ischemia-reperfusion injury though inhibition of miR-2355-3p/Mammalian Sterile20-like kinase 1 (MST1) axis" was retracted in 2026. Reasons: concerns about the data; concerns about the results or conclusions.

Generally, MST1 plays an apoptosis-promoting role in biological function of tissue injury [24,25]. Mitochondrial dysfunction and cardiomyocyte apoptosis are identified as the main cause of I/R injury. Numerous studies indicated MST1 mediates cardiac metabolic damage [26] and autophagy activity [27]. Clinical data showed an upregulation of MST1 in reperfused heart tissue and *in vitro* study illustrated increased MST1 enhanced ROS generation, activated apoptotic pathway, and decreased mitochondrial membrane potential in reperfused cardiomyocytes [28]. Here, our research also compared the fluorescence intensity of ROS between control group and H/R group, the representative images suggested enhanced ROS production in H/R-induced cells. After heart infarction, increased level of MST1 promoted cardiac fibrosis, stimulated inflammatory response and accelerated cell apoptosis, while, inhibition of MST1 prevented the myocardium from chronic post-infarction injury, suggesting MST1 might be a risk factor for post-infarction cardiac injury [29]. Previous study also indicated that activated MST1 attenuated the beneficial effect of melatonin on cell viability and mitochondrial function in cardiomyocyte [30]. Additionally, MST1 was reported to be regulated by different miRNAS in various diseases. miR-199a-5p aggravated abnormal lipid metabolism by targeting MSTI in mice hepatocyte [31]. LncRNA reprogramming (ROR) aggravated cell apoptosis by sponging miR-138 in cardiomyocyte, while miR-138 negatively regulated MST1 expression to mediate H/R-induced injury in H9C2 cells [32]. Sun et al. found miR-486a-5p suppressed MST1 expression to reduce cell death in high-glucose (HG) induced neonatal mouse cardiomyocytes, suggesting miR-486a-5p/MST1 axis was involved in H/R-induced injury [33]. Consistent with previous studies, our research showed elevated MST1 expression in H/R-induced HCMs. Additionally, the further analysis of molecular mechanism demonstrated that circRBMS1 mediated H/R-induced cell injury by targeting miR-2355-3p/MST1. This is the first time to illustrate the regulating mechanism of circRBMS1 and miR-2355-3p/MST1 axis in myocardial I/R injury.

The article "Knockout of circRNA single stranded interacting protein 1 (circRBMS1) played a protective role in myocardial ischemia-reperfusion injury though inhibition of miR-2355-3p/Mammalian Sterile20-like kinase 1 (MST1) axis" was retracted in 2026. Reasons: concerns about the data; concerns about the results or conclusions.

This study also have some limitations. For the mouse model, we only transfected sh-circRBMS1 to the mouse, lacking the co-transfection of miR-2355-3p or MST1 for convincing results. Secondly, some important signal pathways were not discussed. Finally, studies on mitochondrial function and fibrosis in cells could be supplemented. We will supplement these works in future investigation.

## Conclusion

In summary, our study illustrated that increased expression of circRBMS1 and MST1 as well as reduced miR-2355-3p expression was found in cardiac I/R injury. The further study on the molecular mechanism indicated circRBMS1 mediated myocardial I/R injury through miR-2355-3p/MST1 axis. This finding might provide some helpful insights for pathology of I/R injury in heart.

## Supplementary Material

Supplemental Material

## Data Availability

All data can be obtained from the manuscript or from request to the author.
